# Serum IMA and LP-PLA2 Levels in Patients with Coronary Heart Disease and Their Correlation with the Degree of Myocardial Ischaemia and Their Diagnostic Value

This article has been retracted.

**DOI:** 10.1155/2022/1698315

**Published:** 2022-06-11

**Authors:** Likui Zhang, Zipeng Li, Ning Li

**Affiliations:** ^1^Department of Cardiovascular Surgery, Shanxi Bethune Hospital, Shanxi Academy of Medical Sciences, Tongji Shanxi Hospital, Third Hospital of Shanxi Medical University, Taiyuan 030032, China; ^2^Tongji Hospital, Tongji Medical College, Huazhong University of Science and Technology, Wuhan 430030, China; ^3^Department of Vascular Surgery, Beijing Tsinghua Changgung Hospital, Beijing 102200, China; ^4^Department of Cardiovascular Medicine, Shanxi Bethune Hospital, Shanxi Academy of Medical Sciences, Tongji Shanxi Hospital, Third Hospital of Shanxi Medical University, Taiyuan 030032, China

## Abstract

**Purpose:**

To measure serum levels of ischaemia-modified albumin (IMA) and lipoprotein-associated phospholipase A2 (LP-PLA2) in patients with coronary heart disease (CHD) and to analyse their correlation with the degree of myocardial ischaemia and their diagnostic value.

**Methods:**

A sample of 150 patients diagnosed with CHD by coronary angiography in our hospital from March 2019 to September 2021 was taken as the CHD group. The patients were divided into acute myocardial infarction (AMI) group (*n* = 52), unstable angina pectoris (UAP) group (*n* = 54), and stable angina pectoris (SAP) group (*n* = 44) according to the degree of myocardial ischaemia, and then 50 healthy physical examination patients were selected as the health group during the same period. Serum C-reactive protein (CRP), interleukin-6 (IL-6), IMA, and LP-PLA2 levels were measured in each group separately. Multiple ordered logistic regression was used to analyse the factors influencing the degree of myocardial ischaemia in patients with CHD. Pearson correlation was used to analyse the correlation between serum IMA, LP-PLA2 levels and serum CRP, IL-6 levels in CHD patients. The diagnostic value of IMA alone, LP-PLA2 alone, and in combination for CHD was analysed using receiver operating characteristic (ROC) curves.

**Results:**

In terms of serum CRP, IL-6, IMA, and LP-PLA2 levels, the CHD group was higher than the health group, the AMI and UAP groups were higher than the SAP and health groups, and the AMI group was higher than the UAP group (*P* < 0.05). Multiple ordered logistic regression analysis showed that serum CRP, IL-6, IMA, and LP-PLA2 levels were all independent influences on the degree of myocardial ischaemia in patients with CHD (*P* < 0.05). Pearson correlation analysis showed a positive correlation between serum IMA, LP-PLA2 levels and serum CRP, IL-6 levels in CHD patients (*P* < 0.001). The area under curve (AUC) for serum IMA levels to predict myocardial ischaemia in patients with CHD was 0.754 (95% CI: 0.684–0.825), with a sensitivity of 61.3% and specificity of 84.0% when the best cut-off value was 0.453; the AUC for serum LP-PLA2 levels to predict myocardial ischaemia in patients with CHD was 0.747 (95% CI: 0.681–0.813), with a sensitivity of 62.0% and specificity of 82.0% when the optimal cut-off value was 0.440; and the AUC of IMA + LP-PLA2 for predicting myocardial ischaemia in patients with CHD was 0.892 (95% CI: 0.847–0.938), with a sensitivity of 86.7% and specificity of 80.0% when the optimal cut-off value was 0.667. The specificity was 80.0%.

**Conclusions:**

Serum IMA and LP-PLA2 levels are elevated in patients with CHD. Serum IMA and LP-PLA2 levels are closely related to the degree of myocardial ischaemia and its inflammatory level, and the combination of IMA + LP-PLA2 can improve the diagnosis efficacy of myocardial ischaemia in CHD patients.

## 1. Introduction

According to the World Health Organization (WHO) 2018 report, in 2016, approximately 17.9 million people died from cardiovascular diseases worldwide, accounting for 31.4% of global deaths and 44.0% of deaths from chronic noncommunicable diseases (NCDs) [1]. Coronary heart disease (CHD) is a common type of clinical cardiovascular disease, and its morbidity and mortality rates are increasing significantly and tend to be lower in age [2]. It is a heart condition that occurs when there is atherosclerosis of the coronary arteries, the blood vessels that supply the heart muscle, and the lumen is narrowed by more than 50%. The disease can cause incomplete or complete coronary artery obstruction, which in turn triggers temporary or permanent myocardial ischaemia and hypoxia and usually includes clinical pathologies such as stable angina pectoris (SAP) and unstable angina pectoris (UAP) and acute myocardial infarction (AMI) [3]. Unfortunately, the clinical manifestations of early myocardial ischaemia are often vague, diverse, and not easily identifiable. Coupled with the fact that existing myocardial biochemical markers (e.g., creatine kinase isoenzymes, myoglobin, and cardiac troponin) can only be detected after irreversible cell damage and disruption of cell membrane integrity, and that the levels of these markers are not elevated in the blood during short-term and reversible ischaemic episodes, it is of great importance to find an early biochemical diagnostic index of myocardial ischaemia that is cost-effective, rapid, and accurate [4–6].

Ischaemia-modified albumin (IMA) is formed by the modification of alanine, aspartate, histidine, and tonine in the amino terminus of the body's blood albumin under myocardial hypoxia and ischaemia, and it is a sensitive indicator of myocardial ischaemia but cannot distinguish myocardial infarction from myocardial ischaemia [7]. Lipoprotein-associated phospholipase A2 (LP-PLA2) is a phospholipase secreted by inflammatory cells that catalyses the hydrolysis of various oxidised phospholipids and inflammatory factors and is involved in the production of lipid-like proinflammatory substances that have various atherogenic effects [8]. A large number of studies [9, 10] have found that IMA and LP-PLA2 are involved in the development and progression of cardiovascular disease and that their serum change levels are closely related to the inflammatory response and tissue metabolism of patients. However, the clinical application value of the combination of the two in the detection of patients with CHD is yet to be further validated. In this paper, we measured serum IMA and LP-PLA2 levels in CHD patients and analysed their correlation with the degree of myocardial ischaemia and their diagnostic value. The report can be found below.

## 2. Materials and Methods

### 2.1. General Information

A sample of 150 patients diagnosed with CHD by coronary angiography in our hospital from March 2019 to September 2021 was taken as the CHD group. The patients were divided into the AMI group (*n* = 52), the UAP group (*n* = 54), and the SAP group (*n* = 44) according to the degree of myocardial ischaemia. Inclusion criteria: ① all met the American College of Cardiology (ACC)/American Heart Association (AHA) diagnostic criteria [11–13]; ② all with definite vascular lesions confirmed by coronary angiography; and ③ those with complete medical history. Exclusion criteria: ① combined with stroke and other cerebrovascular pathologies; ② combined with congenital heart disease, severe arrhythmia, or other cardiac diseases; ③ combined with peripheral vascular diseases; ④ combined with acute and chronic infectious diseases; ⑤ postcoronary artery bypass grafting or coronary artery stenting; ⑥ combined with autoimmune diseases, malignant tumours, or haematological diseases; ⑦ combined with severe liver and kidney insufficiency; or ⑧ incomplete medical records. And then 50 healthy physical examination patients were selected as the health group during the same period.

### 2.2. Research Methods

#### 2.2.1. Clinical Data Collection

All patients in the CHD group underwent coronary angiography, and the Gensini score was calculated to assess the degree of stenosis and the location of the lesion in the coronary arteries; general medical history (gender, age, body mass index (BMI), smoking history, hypertension, diabetes, stroke history, etc.) and laboratory tests (high-density lipoprotein cholesterol (HDL-C), low-density lipoprotein cholesterol (LDL-C), total cholesterol (TC), triglyceride (TG), fasting blood glucose (FBG), C-reactive protein (CRP), interleukin-6 (IL-6), IMA, LP-PLA2, etc.).

#### 2.2.2. Specimen Collection and Processing

Patients in the CHD group had elbow venous blood collected immediately after admission (FBG was tested using fasting venous blood specimens collected in the early morning of the day after admission), while patients in the health group had fasting elbow venous blood collected in the early morning in accordance with WS/T 225-2016 “Collection and Handling of Blood Specimens for Clinical Chemistry Tests”. 4 ml was collected in a yellow cap vacuum blood tube and centrifuged within 1 h (1000 g, 5 min), and the serum was divided into 2 parts. 1 part was used to measure HDL-C, LDL-C, TC, TG, FBG, CRP, and IL-6 levels within 5 h. The other part was stored in a refrigerator at −80°C for centralised measurement of IMA and LP-PLA2 levels.

#### 2.2.3. Testing Instruments, Methods, and Kits

The testing instrument was the AU5800 fully automatic biochemical analyser (Beckman Coulter, USA). HDL-C and LDL-C (direct method) kits were purchased from Changchun Huili Biotechnology Co. Ltd.; TC, TG, CRP, IL-6, and LP-PLA2 (enzyme linked immunoassay) kits were purchased from Shanghai Ulva Biotechnology Co. Ltd.; the FBG (oxidase method) kit was purchased from Sichuan Mike Biotechnology Co. Ltd.; and the IMA (albumin cobalt binding method) kit was purchased from Beijing Jiuqiang Biotechnology Co. Ltd.

### 2.3. Statistical Methods

Data were processed using SPSS 22.0 software. Categorical variables were expressed as *n* (%), and a *χ*^2^ test was applied. Measures obeying normal distribution were expressed as mean ± standard deviation ($\bar{x}\pm s$), and one-way ANOVA was used for multiple group comparisons, and the *t*-test was used for two-way comparisons. Multiple ordered logistic regression was used to analyse the factors influencing the degree of myocardial ischaemia in CHD patients. Pearson correlation was used to analyse the correlation between serum IMA, LP-PLA2 levels and serum CRP, IL-6 levels in CHD patients. The predictive value of serum LP-PLA2 and IMA levels for the development of myocardial ischaemia in patients with CHD was analysed using receiver operating characteristic (ROC) curves. The test level was *α* = 0.05, and *P* < 0.05 was considered a statistically significant difference.

## 3. Results

### 3.1. Comparison of General Information between the CHD Group and the Health Group

There was no statistical difference between the CHD group and the health group in terms of gender and age (*P* > 0.05). There was a statistical difference between the CHD group and the health group in terms of smoking history, hypertension, diabetes, stroke history, and HDL-C, BMI, LDL-C, TC, TG, and FBG levels (*P* < 0.05) (Table 1).

### 3.2. Comparison of Serum CRP, IL-6, IMA, and LP-PLA2 Levels between the Observation and Health Groups

The serum CRP, IL-6, IMA, and LP-PLA2 levels were higher in the CHD group than in the health group (*P* < 0.05) (Figures 1–4).

### 3.3. Comparison of Serum CRP, IL-6, IMA, and LP-PLA2 Levels between the Groups

The serum levels of CRP, IL-6, IMA, and LP-PLA2 were higher in the AMI and UAP groups than in the SAP and health groups, as well as in the AMI group than in the UAP group (*P* < 0.05). (Figures 5–8).

### 3.4. Multivariate Ordered Logistic Regression Analysis of Factors Influencing the Degree of Myocardial Ischaemia in Patients with CHD

Serum CRP, IL-6, IMA, and LP-PLA2 levels were used as independent variables, and the degree of myocardial ischaemia was used as the dependent variable in a multivariate ordered logistic regression analysis. The results showed that serum CRP, IL-6, IMA, and LP-PLA2 levels were all independent influences on the degree of myocardial ischaemia in patients with CHD (*P* < 0.05) (Tables 2 and 3).

### 3.5. Correlation of Serum IMA, LP-PLA2 Levels with Serum CRP, and IL-6 Levels in Patients with CHD

Pearson correlation analysis showed that serum IMA levels in CHD patients were positively correlated with CRP (*r* = 0.751) and IL-6 (*r* = 0.772) levels (*P* < 0.001) and that serum LP-PLA2 levels were positively correlated with CRP (*r* = 0.790) and IL-6 (*r* = 0.814) levels (*P* < 0.001) (Table 4).

### 3.6. Predictive Value of Serum IMA and LP-PLA2 Levels for the Development of Myocardial Ischaemia in Patients with CHD

The area under curve (AUC) for serum IMA levels to predict myocardial ischaemia in patients with CHD was 0.754 (95% CI: 0.684–0.825), with a sensitivity of 61.3% and specificity of 84.0% when the best cut-off value was 0.453; the AUC for serum LP-PLA2 levels to predict myocardial ischaemia in patients with CHD was 0.747 (95% CI: 0.681–0.813), with a sensitivity of 62.0% and specificity of 82.0% when the optimal cut-off value was 0.440; and the AUC of IMA + LP-PLA2 for predicting myocardial ischaemia in patients with CHD was 0.892 (95% CI: 0.847–0.938), with a sensitivity of 86.7% and specificity of 80.0% when the optimal cut-off value was 0.667. The specificity was 80.0% (Table 5, Figure 9).

## 4. Discussion

Myocardial ischaemia is a pathological state in which the heart has reduced blood perfusion, reduced oxygen supply, and abnormal myocardial energy metabolism that do not support the normal work of the heart. Data [14] show that coronary artery disease is the most common cause of myocardial ischaemia, which usually includes SAP, UAP, AMI, and other disease types and is part of a continuous disease spectrum. Clinical practice [15] has shown that when the disease is in the UAP stage, myocardial cells have not yet developed ischaemic necrosis and that timely detection and effective treatment during this period can minimise myocardial cell damage and improve the patient's prognosis. This shows that myocardial ischaemia, if rapidly corrected, has a low impact on the long-term prognosis; otherwise, death may result from eventual myocardial infarction, fatal arrhythmias, or pump failure.

It is well known that inflammatory responses are present throughout the development and progression of coronary artery disease. CRP and IL-6 are the most common inflammatory factors. The former is a sensitive indicator of tissue damage and inflammatory response in the body; and the latter activates monocytes and promotes their adhesion and chemotaxis to vascular smooth muscle, prompting it to proliferate and migrate, and it also induces macrophages to migrate towards plaques, participating in their formation and accelerating their rupture [16, 17]. In addition, IMA is an albumin produced as a result of local structural changes in the flow of human serum albumin through ischaemic tissues. IMA has been clinically found to be involved in the process of myocardial injury, but the mechanism of action has not been fully defined. It is now generally accepted that it is closely related to various phenomena, such as activation of inflammatory responses, free radical damage, acidosis, and disruption of calcium pumps, and that IMA can be dramatically increased when the body is ischaemic and hypoxic [17]. LP-PLA2 is a specific vascular inflammatory mediator produced mainly by lymphocytes and macrophages. Studies [18] suggest that elevated levels may mediate an enzymatic response to inflammatory factors that contribute to the rupture and dislodgement of atheromatous plaques, which in turn can lead to myocardial infarction and aggravate the progression of the disease. In this result, in terms of serum CRP, IL-6, IMA, and LP-PLA2 levels, the CHD group was higher than the health group, the AMI and UAP groups were higher than the SAP and health groups, and the AMI group was higher than the UAP group (*P* < 0.05). Further multivariate ordered logistic regression analysis showed that serum CRP, IL-6, IMA, and LP-PLA2 levels were all independent influences on the degree of myocardial ischaemia in patients with CHD (*P* < 0.05). This suggests that serum levels of CRP, IL-6, IMA, and LP-PLA2 are elevated in patients with CHD and that their levels tend to be highly expressed as the patients' myocardial ischaemia increases. In the results, Pearson correlation analysis showed a positive correlation between serum IMA, LP-PLA2 levels and CRP, IL-6 levels in CHD patients (*P* < 0.001). It was suggested that serum IMA and LP-PLA2 levels in CHD patients were positively correlated with the degree of myocardial ischaemia and serum inflammation levels of the patients. The reason for this is that LP-PLA2, through its hydrolysis products, can upregulate the expression of endothelial cell adhesion molecules to induce inflammatory factor activation, which in turn activates more monocytes/macrophages into the plaque and also induces matrix metalloproteinases to be secreted by the atherosclerotic plaque, leading to degradation of the plaque fibrous cap and glial matrix, resulting in plaque detachment and vascular blockage, further aggravating ischaemia and hypoxia symptoms. This leads to a rapid increase in serum IMA levels, and inflammatory cells in the atherosclerotic plaque can then produce more LP-PLA2, thus creating a vicious cycle that leads to a self-reinforcing inflammatory response and accelerates arterial vascular disease [19].

Abnormal expression of serum IMA and LP-PLA2 levels in patients with CHD has been reported [20]. Therefore, monitoring changes in CHD during its onset and progression may be a key breakthrough for early detection of myocardial ischaemia and improving the prognosis of CHD patients. The concentration of IMA in peripheral blood rises rapidly 5–10 minutes after myocardial ischaemia and continues to rise during the ischaemic process. Elevated serum levels of IMA can be detected earlier than other markers of myocardial injury such as creatine kinase isoenzymes, so the diagnosis of myocardial ischaemia can be made in time before myocardial necrosis by measuring serum IMA levels [21]. Besides, 70% of Lp-PLA2 hydrolysed and oxidatively modified low-density lipoprotein (ox-LDL) particles produce metabolites such as haemolytic lecithin and oxidised free fatty acids, which cause endothelial dysfunction, necrosis, and apoptosis through an inflammatory chain reaction, leading to atherosclerosis progression and plaque instability [22]. Mechanistically, elevated Lp-PLA2 levels could also be used as an early biochemical predictor of the degree of myocardial ischaemia. In this result, the AUC for IMA and LP-PLA2 to predict myocardial ischaemia in CHD patients was 0.754 and 0.747, respectively; and the AUC for IMA + LP-PLA2 combination to predict myocardial ischaemia in CHD patients was 0.892. It is suggested that the diagnostic value of the IMA + LP-PLA2 test in predicting myocardial ischaemia in CHD patients is higher than that of the single test. The clinical assessment of patients' conditions can be based on the results of the two tests, and corresponding therapeutic measures can be taken to improve patients' prognosis and quality of life.

Serum IMA and LP-PLA2 levels are elevated in patients with CHD. Serum IMA and LP-PLA2 levels are closely related to the degree of myocardial ischaemia and its inflammatory level, and the combination of IMA + LP-PLA2 can improve the diagnosis efficacy of myocardial ischaemia in CHD patients.

## Figures and Tables

**Figure 1:** Serum CRP level (mg/L).

**Figure 2:** Serum IL-6 level (*μ*g/L).

**Figure 3:** Serum IMA level (U/ml). Note: ^*∗*^ is *P* < 0.05 compared with the CHD group.

**Figure 4:** Serum LP-PLA2 level (U/L). Note: ^*∗*^ is *P* < 0.05 compared with the CHD group.

**Figure 5:** Serum CRP level (mg/L).

**Figure 6:** Serum IL-6 level (*μ*g/L).

**Figure 7:** Serum IMA level (U/ml). Note: ^*∗*^ is *P* < 0.05 compared with SAP group and health group, and^∧^is *P* < 0.05 compared with UAP group.

**Figure 8:** Serum LP-PLA2 level (U/L). Note: ^*∗*^ is *P* < 0.05 compared with SAP group and health group, and ^ is *P* < 0.05 compared with UAP group.

**Figure 9:** ROC curves of serum LP-PLA2 and IMA levels predicting myocardial ischaemia in patients with CHD.

**Table 1:** Comparison of general information between the CHD group and the health group.

Indicators	CHD group (*n* = 150)	Health group (*n* = 50)	*χ* ^2^/*t*	*P*
Male/female (cases)	79/71	30/20	0.813	0.367
Smoking history (case)	82	14	10.684	0.001
Hypertension (case)	91	0	55.658	<0.001
Diabetes (case)	51	0	22.819	<0.001
Stroke history (case)	22	0	8.240	0.004
Age (years)	60.09 ± 6.82	58.40 ± 7.40	0.1485	0.139
BMI (kg/m^2^)	25.44 ± 2.27	22.45 ± 2.14	8.179	<0.001
HDL-C (mmol/L)	1.04 ± 0.24	1.34 ± 0.26	7.495	<0.001
LDL-C (mmol/L)	2.64 ± 1.01	2.20 ± 0.58	2.92	0.004
TC (mmol/L)	4.70 ± 1.10	4.26 ± 0.90	2.556	0.011
TG (mmol/L)	1.52 ± 0.47	1.26 ± 0.37	3.559	0.001
FBG (mmol/L)	6.79 ± 1.57	5.76 ± 0.43	4.575	<0.001

**Table 2:** Variable assignment table.

Variables	Assignment
CRP	Continuous variable
IL-6	Continuous variable
IMA	Continuous variable
LP-PLA2	Continuous variable
Myocardial ischaemia degree	SAP = 1, UAP = 2, AMI = 3

**Table 3:** Multivariate ordered logistic regression analysis of factors influencing the degree of myocardial ischaemia in patients with CHD.

Variables	*β*	SE	Wald	OR (95% CI)	*P*
CRP	1.425	0.457	4.167	4.158 (1.698, 10.183)	0.041
IL-6	0.973	0.414	5.335	2.646 (1.175, 5.956)	0.021
IMA	0.954	0.212	5.617	2.596 (1.713, 3.933)	0.018
LP-PLA2	0.762	0.214	5.717	2.143 (1.409, 3.259)	0.017

**Table 4:** Correlation of serum IMA, LP-PLA2 levels with serum CRP, IL-6 levels in patients with CHD.

Indicators	CRP		IL-6	
	*r*	*P*	*r*	*P*
IMA	0.751	<0.001	0.772	<0.001
LP-PLA2	0.790	<0.001	0.814	<0.001

**Table 5:** Predictive value of serum IMA and LP-PLA2 levels for the development of myocardial ischaemia in patients with CHD.

Indicators	AUC	Approaching 95% confidence interval		Optimal cut-off value	Sensitivity %	Specificity %
		Lower limit	Upper limit			
IMA	0.754	0.684	0.825	0.453	61.3	84.0
LP-PLA2	0.747	0.681	0.813	0.440	62.0	82.0
IMA + LP-PLA2	0.892	0.847	0.938	0.667	86.7	80.0

## Data Availability

All data in the submitted article used or analysed can be obtained from the respective authors.
